# Anticollision Decision and Control of UAV Swarm Based on Intelligent Cognitive Game

**DOI:** 10.1155/2022/6398039

**Published:** 2022-08-11

**Authors:** Huan Zhou, Yintong Li, Tong Han

**Affiliations:** Aviation Engineering School, Air Force Engineering University, Xi'an, China

## Abstract

UAV swarm anticollision system is very important to improve the flight safety of the whole swarm formation, while the existing system design methods are still insufficient in realizing autonomous and cooperative anticollision. Based on the cognitive game theory, an intelligent decision-making and control method for UAV swarm anticollision is designed. Firstly, by using the idea of swarm intelligence, basic flight behaviors of UAV swarm are defined as five basic flight rules, such as cohesion, following, self-guidance, dispersion, and alliance. Further, the cognitive security domain of UAV swarm is constructed by setting the overall anticollision rules of the swarm and the anticollision rules of individual members. On this basis, the anticollision problem of UAV swarm is transformed into a game problem involving two parties, and the solution method of decision and control strategy set is proposed. Finally, the stability of anticollision decision and control method is proved through eigenvalue theory. The simulation results show that the method proposed in this paper can effectively realize the autonomous cooperative anticollision of UAV swarm and also has good algorithm real-time solution ability while ensuring flight safety.

## 1. Introduction

The operational mission requirements such as cooperative reconnaissance, cooperative tracking, and cooperative strike faced by UAV autonomous cooperation determine that its operational use mode is multi-aircraft swarm system [1, 2]. The application of swarm enables UAV to cover a wide area in less time in reconnaissance, search, and rescue tasks, which greatly improves the use efficiency of UAV. However, the increase in the number and density of space UAVs has also brought great challenges to flight safety at the same time [3, 4]. Autonomous flight and evasion control of swarm system has become an urgent problem to be solved.

For a swarm system, there are currently two main control methods: leader follower [5–7] and behavior control [8–10]. The idea of the leader follower method is to introduce a leader and use the distributed control method to control other followers in the swarm, so that the state (such as speed) of all followers gradually follows the leader and finally achieves consistency. In reference [7], considering system noise and time delay, the coordination problem of second-order definite topology multi-agent system with leader is studied by using control theory. Behavior control mainly draws lessons from the idea of swarm intelligence, designs the motion behavior of swarm system based on evolutionary mechanism, and has adaptive ability through certain evolution and development. Among them, literature [8] established a two-dimensional in-plane swarming algorithm based on the UAV model of constant speed and inclined turning. The algorithm includes two basic rules: alliance and cohesion. A great contribution of this paper is to prove that the weight of the rules will determine the flight behavior of the swarm.

At present, the commonly used swarm system avoidance control methods mainly include geometric vectors [11, 12], artificial potentials [13–15], and model predictive control (MPC) [16–18]. Geometric vector method often has no speed limit on the internal members of the swarm system, which is not allowed by UAV, so it is mainly used in the control of ground robot. The artificial potential field method regards the motion of UAV as the result of the interaction of attraction and repulsion, but this method is easy to fall into local minimum. One of the main advantages of model predictive control is that it can effectively solve the problems of constraints or high dimension of the system, but the amount of system calculation increases significantly with the increase of the number of swarm members, which is difficult to meet the real-time requirements [19].

In order to overcome the shortcomings of the above methods, inspired by the idea of swarm intelligence in reference [8], this paper studies the UAV swarm flight and evasion control method based on rules. Firstly, the basic flight rules of UAV members in the swarm are defined to control the normal level flight of the swarm. On this basis, the evasion action is regarded as another flight rule of the swarm. By setting the corresponding rule weight coefficient, two mechanisms of the whole and members are established for swarm evasion guidance and control. Simulation results show that the proposed method can effectively realize swarm flight and evasion, and has good real-time performance.

## 2. Basic Flight Behavior Rules of Swarm

In order to control the normal flight and formation reconstruction of the swarm system, using the idea of swarm intelligence for reference, the basic flight rules of UAV members in the swarm system are abstracted as cohesion, following, self-guidance, dispersion, and alliance.

### 2.1. Swarm Intelligence

Swarm intelligence is a computing technology based on the behavior law of biological groups. There are two main algorithms in this theoretical research field: ant colony algorithm [20] (ACA) and particle swarm optimization [21] (PSO). In the field of computer science and application research, ant colony algorithm is a probability theory method to solve mathematical problems. It uses graph theory to find optimization and optimal path. Dr. Kennedy and Dr. Eberhart first proposed the particle swarm optimization algorithm in 1995, inspired by the social behaviors such as predation of birds and fish. PSO algorithm is similar to genetic algorithm in evolutionary computation, but different from genetic algorithm, it has no evolutionary mechanism such as crossover and mutation.

At present, because ant colony algorithm and particle swarm optimization algorithm have many advantages, they are widely used in research and application fields. At the same time, swarm intelligence method [22] is also gradually rising. Based on the traditional swarm intelligence algorithm, this method aims to realize the distributed intelligent cooperative control of multirobots, multiagents, and multiaircraft platforms. Swarm intelligence algorithm regards each agent/member in the swarm system as an individual in the biological system. Individuals with the same or similar characteristics form a new swarm. The interaction between swarm individuals or swarms adopts the influence mechanism of traditional swarm intelligence algorithm. In this way, the swarm intelligent algorithm will have the characteristics of simple algorithm, easy to meet real time, high degree of intelligence, and good robustness.

### 2.2. Basic Flight Rules for Internal Members of the Swarm System

The geometric parameters of single and two UAV members in the swarm system are shown in Figures 1 and 2 respectively.

According to the six degree-of-freedom motion equations of UAV [23], the partial velocities of each member in the swarm system in the three axes in the geographic coordinate system are $\dot{x},\dot{y},\dot{z}$, respectively:

(1) $$\begin{array}{c} \dot{x}=V\;\cos\;\theta \;\cos\;\psi , \end{array}$$

(2) $$\begin{array}{c} \dot{y}=V\;\cos\;\theta \;\sin\;\psi , \end{array}$$

(3) $$\begin{array}{c} \dot{z}=V\;\sin\;\theta , \end{array}$$

where *x*, *y*, *z* are the three-axis coordinates of the UAV, *ψ*, *θ* are the track deflection angle and track inclination angle of the UAV, *V* is the flight speed scalar of the UAV, and the two angular speeds $\dot{\psi },\dot{\theta }$ of the UAV are expressed by the following formula:

(4) $$\begin{array}{c} \dot{\psi }=\frac{\kappa_{\psi }}{V\;\cos\;\theta }, \end{array}$$

(5) $$\begin{array}{c} \dot{\theta }=\frac{\kappa_{\theta }}{V}, \end{array}$$

where *κ*_*ψ*_ and *κ*_*θ*_ are the acceleration term coefficients of angular velocity.

In Figure 2, *ψ*^*r*^, *θ*^*r*^, *R*^*r*^ are the relative track deflection angle, relative track inclination angle, and relative distance on the sight distance of two UAV members, respectively. Make the angular velocity $\overset{\cdot }{\psi },\overset{\cdot }{\theta }$ of UAVs in the swarm proportional to the deviation between the expected attitude angle and the current attitude angle:

(6) $$\begin{array}{c} \kappa_{\psi }=k_{1}\Delta \psi_{\text{d}}, \end{array}$$

(7) $$\begin{array}{c} \kappa_{\theta }=k_{2}\Delta \theta_{\text{d}}, \end{array}$$

(8) $$\begin{array}{c} \Delta \psi_{\text{d}}=\psi_{\text{d}}-\psi , \end{array}$$

(9) $$\begin{array}{c} \Delta \theta_{\text{d}}=\theta_{\text{d}}-\theta , \end{array}$$

where *k*_1_,  *k*_2_ are proportional constants, *ψ*_d_, *θ*_d_ are the expected track deflection angle and the expected track inclination angle, respectively, *ψ*, *θ* are the current track deflection angle and the current track inclination angle, respectively, and Δ*ψ*_d_, Δ*θ*_d_ are the deviation between the expected track deflection angle and the current track deflection angle and the deviation between the expected track inclination angle and the current track inclination angle, respectively. Among them, the desired attitude angle of UAV is calculated by the flight rules of UAV swarm. When the number of effective flight rules of UAV is greater than 1, the expected attitude angle deviation can be obtained from the following formula:

(10) $$\begin{array}{c} \Delta \psi_{\text{d}}=\tau_{1}\left(\psi_{{\text{d}}_{1}}-\psi \right)+\tau_{2}\left(\psi_{{\text{d}}_{2}}-\psi \right)+\cdots +\tau_{n}\left(\psi_{{\text{d}}_{n}}-\psi \right), \end{array}$$

(11) $$\begin{array}{c} \Delta \theta_{\text{d}}=\tau_{1}\left(\theta_{{\text{d}}_{1}}-\theta \right)+\tau_{2}\left(\theta_{{\text{d}}_{2}}-\theta \right)+\cdots +\tau_{n}\left(\theta_{{\text{d}}_{n}}-\theta \right), \end{array}$$

where *ψ*_d_1__, *ψ*_d_2__,…, *ψ*_d_*n*__ and *θ*_d_1__, *θ*_d_2__,…, *θ*_d_*n*__ are the expected track deflection angle and expected track inclination under the action of the first to n-th flight rules, respectively, and *τ*_1_, *τ*_2_,…, *τ*_*n*_ is the weight corresponding to the first to n-th flight rules.

For the i-th UAV member in the swarm system, the basic flight rules are abstracted as the following five.

*Cohesion*. The cohesion feature can make the internal members of the swarm system close to each other to maintain the swarm formation. Each UAV member in the swarm approaches the UAV within its detection distance, that is, the expected velocity vector of the UAV points to the centroids of several UAV members within its detection distance *ρ*. Suppose that the i-th UAV member in the swarm can detect *n*_*i*_ UAV members; (*X*_*i*_*M*__, *Y*_*i*_*M*__, *Z*_*i*_*M*__) is the average centroid coordinate of *n*_*i*_ UAV members, and (*X*_*i*_, *Y*_*i*_, *Z*_*i*_) is the centroid coordinate of the *i*-th UAV member; then under this flight rule, the expected track deflection angle *ψ*_d*i*_*M*__ and expected track inclination angle *θ*_d*i*_*M*__ of the *i*-th UAV member are, respectively,

(12) $$\begin{array}{c} \psi_{\text{d}i_{M}}=\arctan\left(\frac{Y_{i_{M}}-Y_{i}}{X_{i_{M}}-X_{i}}\right), \end{array}$$

(13) $$\begin{array}{c} \theta_{\text{d}i_{M}}=\arctan\left(\frac{Z_{i_{M}}-Z_{i}}{\sqrt{{\left(X_{i_{M}}-X_{i}\right)}^{2}+{\left(Y_{i_{M}}-Y_{i}\right)}^{2}}}\right). \end{array}$$

*Follow*. The follow feature enables each member in the swarm system to follow the other two members. One member is closest to the UAV member, and the other member is randomly selected within the system. Let (*X*_*i*_*L*__, *Y*_*i*_*L*__, *Z*_*i*_*L*__) be the centroid coordinate of the UAV nearest to the UAV member and (*X*_*i*_*R*__, *Y*_*i*_*R*__, *Z*_*i*_*R*__) be the centroid coordinate of the randomly selected UAV; then under this flight rule, the expected track deflection angle *ψ*_d*i*_*F*__ and expected track inclination angle *θ*_d*i*_*F*__ of the i-th UAV member can be obtained by the following formula:

(14) $$\begin{array}{c} \psi_{\text{d}i_{L}}=\arctan\left(\frac{Y_{i_{L}}-Y_{i}}{X_{i_{L}}-X_{i}}\right), \end{array}$$

(15) $$\begin{array}{c} \theta_{\text{d}i_{L}}=\arctan\left(\frac{Z_{i_{L}}-Z_{i}}{\sqrt{{\left(X_{i_{L}}-X_{i}\right)}^{2}+{\left(Y_{i_{L}}-Y_{i}\right)}^{2}}}\right), \end{array}$$

(16) $$\begin{array}{c} \psi_{di_{R}}=\arctan\left(\frac{Y_{i_{R}}-Y_{i}}{X_{i_{R}}-X_{i}}\right), \end{array}$$

(17) $$\begin{array}{c} \theta_{di_{R}}=\arctan\left(\frac{Z_{i_{R}}-Z_{i}}{\sqrt{{\left(X_{i_{R}}-X_{i}\right)}^{2}+{\left(Y_{i_{R}}-Y_{i}\right)}^{2}}}\right), \end{array}$$

(18) $$\begin{array}{c} \psi_{\text{d}i_{F}}=\frac{\psi_{\text{d}i_{L}}+\psi_{\text{d}i_{R}}}{2}, \end{array}$$

(19) $$\begin{array}{c} \theta_{\text{d}i_{F}}=\frac{\theta_{\text{d}i_{L}}+\theta_{\text{d}i_{R}}}{2}. \end{array}$$

*Homing*. The homing feature enables swarm system members to track specific signals to fly to a specified area. Let (*X*_*i*_*I*__, *Y*_*i*_*I*__, *Z*_*i*_*I*__) be the coordinate where the tracking signal is located; then under this flight rule, the expected track deflection angle *ψ*_d*i*_*I*__ and expected track inclination angle *θ*_d*i*_*I*__ of the i-th UAV member are, respectively,

(20) $$\begin{array}{c} \psi_{\text{d}i_{I}}=\arctan\left(\frac{Y_{i_{I}}-Y_{i}}{X_{i_{I}}-X_{i}}\right), \end{array}$$

(21) $$\begin{array}{c} \theta_{\text{d}i_{I}}=\arctan\left(\frac{Z_{i_{I}}-Z_{i}}{\sqrt{{\left(X_{i_{I}}-X_{i}\right)}^{2}+{\left(Y_{i_{I}}-Y_{i}\right)}^{2}}}\right), \end{array}$$

*Dispersion*. The dispersion feature can keep enough safe distance between members in the swarm, that is, ensure that the flight interval between any two members does not exceed *s*_min_. Therefore, each UAV member flies in the opposite direction of other UAVs in the swarm to prevent UAVs from getting too close. Let (*X*_*i*_*S*__, *Y*_*i*_*S*__, *Z*_*i*_*S*__) be the average centroid coordinate of the *i*-th UAV whose distance from the UAV member is less than *s*_min_; then under this flight rule, the expected track deflection angle *ψ*_d*i*_*S*__ and expected track inclination angle *θ*_d*i*_*S*__ of the *i*-th UAV member are, respectively,

(22) $$\begin{array}{c} \psi_{\text{d}i_{S}}=-\arctan\left(\frac{Y_{i_{S}}-Y_{i}}{X_{i_{S}}-X_{i}}\right), \end{array}$$

(23) $$\begin{array}{c} \theta_{\text{d}i_{S}}=\arctan\left(\frac{Z_{i_{S}}-Z_{i}}{\sqrt{{\left(X_{i_{S}}-X_{i}\right)}^{2}+{\left(Y_{i_{S}}-Y_{i}\right)}^{2}}}\right). \end{array}$$

*Alliance*. The alliance feature can keep the internal members of the swarm system in a certain order and ensure the flight of the swarm system as a whole. Each UAV member flies in the direction of the average velocity vector of the UAV within its detection range. Under this flight rule, the expected track deflection angle *ψ*_d*i*_*A*__ and expected track inclination angle *θ*_d*i*_*A*__ of the *i*-th UAV member are, respectively,

(24) $$\begin{array}{c} \psi_{\text{d}i_{A}}=\left(\frac{1}{n_{i}}\right)\sum_{j=1}^{n_{i}}\left(\psi_{\text{d}j_{A}}\right), \end{array}$$

(25) $$\begin{array}{c} \theta_{\text{d}i_{A}}=\left(\frac{1}{n_{i}}\right)\sum_{j=1}^{n_{i}}\left(\theta_{\text{d}j_{A}}\right). \end{array}$$

## 3. Cognitive Security Domain for Swarm Anticollision

The swarm collaboration adopts a distributed mechanism. Each member of the system uses airborne sensors to detect the unknown environment. The members communicate based on the global fully connected topology to realize information sharing. When sensing the threat of obstacles, they can evade in real time and independently. It is assumed that accurate environmental state information has been obtained after fusion filtering of sensor data. Based on the basic flight rules of the internal members of the swarm system, the swarm evasion action is also regarded as the flight rules of the internal members of the swarm. Similarly, under the evasion flight rules, the expected track deflection angle and expected track inclination angle of the *i*-th UAV member are *ψ*_d*i*_*E*__ and *θ*_d*i*_*E*__, respectively. Therefore, the swarm system avoiding collaborative control can be described as follows.

By calculating such a desired track deflection angle *ψ*_d*i*_ and desired track inclination angle *θ*_d*i*_ (for the *i*-th UAV member in a swarm), Δ*ψ*_d*i*_ and Δ*θ*_d*i*_ are obtained, and the guidance command is transmitted to the autopilot of the corresponding UAV. Under the action of the flight control system, it can ensure that no member in the swarm system will collide with other members in the swarm or other threats outside the swarm, so as to realize safe flight.

The above calculation formulas of Δ*ψ*_d*i*_ and Δ*θ*_d*i*_ are as follows:

(26) $$\begin{array}{c} \Delta \psi_{\text{d}i}=\tau_{i_{M}}\left(\psi_{\text{d}i_{M}}-\psi \right)+\tau_{i_{F}}\left(\psi_{\text{d}i_{F}}-\psi \right)+\tau_{i_{I}}\left(\psi_{\text{d}i_{I}}-\psi \right)\\ +\tau_{i_{S}}\left(\psi_{\text{d}i_{S}}-\psi \right)+\tau_{i_{A}}\left(\psi_{\text{d}i_{A}}-\psi \right)+\tau_{i_{E}}\left(\psi_{\text{d}i_{E}}-\psi \right), \end{array}$$

(27) $$\begin{array}{c} \Delta \theta_{\text{d}i}=\tau_{i_{M}}\left(\theta_{\text{d}i_{M}}-\theta \right)+\tau_{i_{F}}\left(\theta_{\text{d}i_{F}}-\theta \right)+\tau_{i_{I}}\left(\theta_{\text{d}i_{I}}-\theta \right)\\ +\tau_{i_{S}}\left(\theta_{\text{d}i_{S}}-\theta \right)+\tau_{i_{A}}\left(\theta_{\text{d}i_{A}}-\theta \right)+\tau_{i_{E}}\left(\theta_{\text{d}i_{E}}-\theta \right). \end{array}$$

By setting different weights of flight rules, swarm evasion cooperative control is divided into two decision-making mechanisms: overall evasion mechanism and member evasion mechanism. In the first mechanism, UAV swarm as a whole can avoid collision threat. In the second mechanism, the UAV swarm can avoid the collision threat through the flight behavior of each member.

### 3.1. Overall Avoidance Mechanism

In the overall evasion mechanism, the UAV swarm as a whole, in order to ensure that the internal members of the swarm do not separate during the evasion process, the weight of the cohesive flight rules of the UAV swarm is large. Under the action of avoiding flight rules, the expected track deflection angle of the i-th UAV member in the swarm is

(28) $$\begin{array}{c} \psi_{\text{d}i_{E}}=f_{1}\left(\frac{\pi }{2}\right)+\psi_{i}, \end{array}$$

where *f*_1_ is the transformation function of track deflection direction in the horizontal plane set to complete evasion. Let (*X*_*i*_*T*__, *Y*_*i*_*T*__, *Z*_*i*_*T*__) be the average centroid coordinates of all collision threats outside the swarm at the detection distance of the i-th UAV member, then *f*_1_(*x*) is expressed as

(29) $$\begin{array}{c} f_{1}\left(x\right)=\left\{\begin{array}{c} -x,\frac{\pi }{4}<\psi_{i}\leq \frac{3\pi }{4}\text{and }X_{i}\geq X_{i_{T}}\\ x,\frac{\pi }{4}\leq \psi_{i}<\frac{3\pi }{4}\text{and }X_{i}<X_{i_{T}}\\ x,\frac{5\pi }{4}<\psi_{i}\leq \frac{7\pi }{4}\text{and }X_{i}\geq X_{i_{T}}\\ -x,\frac{5\pi }{4}\leq \psi_{i}<\frac{7\pi }{4}\text{and }X_{i}<X_{i_{T}}\\ -x,\frac{3\pi }{4}<\psi_{i}\leq \frac{5\pi }{4}\text{and }Y_{i}\geq Y_{i_{T}}\\ x,\frac{3\pi }{4}\leq \psi_{i}<\frac{5\pi }{4}\text{and }Y_{i}<Y_{i_{T}}\\ x,\left(\frac{7\pi }{4}<\psi_{i}\leq 2\pi \;\mathrm{or}\;0<\psi_{i}\leq \frac{\pi }{4}\right)\text{and}Y_{i}\geq Y_{i_{T}}\\ -x,\left(\frac{7\pi }{4}\leq \psi_{i}<2\pi \;\mathrm{or}\;0\leq \psi_{i}<\frac{\pi }{4}\right)\text{and}Y_{i}<Y_{i_{T}} \end{array}\right.. \end{array}$$

According to equation (29), the overall avoidance mechanism can be explained as follows: when the distance between the swarm and the collision threat gradually increases, the swarm flies along the pre-planned track; when the swarm and the collision threat gradually approach and the distance between them is less than a certain value, according to equation (28), the swarm system performs avoidance cooperative control as a whole. The transformation of track deflection angle of each UAV member depends on the position coordinate relationship between the UAV and the collision threat.

Similarly, in the overall avoidance mechanism, the expected track inclination of the i-th UAV member in the swarm is

(30) $$\begin{array}{c} \theta_{AVi}=f_{2}\left(\frac{\pi }{2}\right)+\theta_{i}, \end{array}$$

where *f*_2_ is the transformation function of track inclination direction in the vertical plane set to complete evasion and *f*_2_(*x*) is expressed as

(31) $$\begin{array}{c} f_{2}\left(x\right)=\left\{\begin{array}{cc} x, & Z_{i}\geq Z_{i_{T}},\\ -x, & Z_{i}<Z_{i_{T}}. \end{array}\right. \end{array}$$

For the *i*-th UAV member, the weight of circumvention rule is defined as follows:

(32) $$\begin{array}{c} \tau_{i_{E}}=\left\{\begin{array}{cc} 1, & \left\|P_{i}-P_{\rho i}\right\|\leq \rho_{c},\\ 0, & \left\|P_{i}-P_{\rho i}\right\|>\rho_{c}, \end{array}\right. \end{array}$$

where **P**_*i*_=(*X*_*i*_, *Y*_*i*_, *Z*_*i*_), **P**_*ρi*_=(*X*_*i*_*T*__, *Y*_*i*_*T*__, *Z*_*i*_*T*__), *ρ*_*c*_ is defined as the evasion distance of UAV members; that is, the evasion control is carried out only when the distance between two centroids is less than *ρ*_*c*_.

### 3.2. Member Avoidance Mechanism

In the member evasion mechanism, the control method is similar to the overall evasion mechanism, except for the weight of flight rules. At the same time, the extended distance *ρ*_*e*_ is defined based on the available detection distance *ρ* and evasion distance *ρ*_*c*_ of the sensor. The three distances defined in this paper have the following relationship: *ρ*_*c*_ < *ρ*_*e*_ < *ρ*.

Set the minimum interval *s*_min_′ between any two UAV members in the same swarm to

(33) $$\begin{array}{c} s_{\min}^{\prime }=\left\{\begin{array}{cc} s_{1}, & \left\|P_{i}-P_{\rho i}\right\|\leq \rho_{e},\\ s_{2}, & \left\|P_{i}-P_{\rho i}\right\|>\rho_{e}, \end{array}\right. \end{array}$$

where *s*_1_ > *s*_2_.

Then, the member avoidance mechanism can be explained as follows: when the collision threat is within the extended distance *ρ*_*e*_ of any UAV member in the swarm system, the value of *s*_min_′ increases from *s*_2_ to *s*_1_, so that the swarm system can allow the collision threat to pass through the swarm during the avoidance process. When the collision threat enters the swarm and is within the avoidance distance *ρ*_*c*_ of its internal members, the avoidance decision will be made, and the rule weight, expected track deflection angle, and expected track inclination angle can be obtained from equations (28)–(32). Under this mechanism, the cohesion weight *τ*_*i*_*M*__ is reduced, so that the distance expansion between members in the swarm system can be better realized.

### 3.3. Cognitive Security Domain

The autonomous anticollision decision and control of UAV swarm include anticollision and separation guarantee, that is, to keep any member in the swarm outside the area surrounding each member adjacent to it. For the sake of safety, assuming that only UAV maneuvers to avoid collision, the above area is defined as the safety area of UAV, and the safety goal is to ensure that no other UAV penetrates the area. The exact mathematical expression of cognitive security domain is given below.

Let **z**(*t*) ∈ *ℝ*^d^ represent the state vector of two conflicting UAVs at any time *t* > 0. It is assumed that its variation law can be described by a differential equation:

(34) $$\begin{array}{c} \left\{\begin{array}{c} \dot{z}\left(s\right)=f\left(z\left(s\right),s,u\left(s\right),r\left(s\right)\right),\forall s\in \left[0,t\right],\\ z\left(0\right)=z_{0}, \end{array}\right. \end{array}$$

where **u**(*·*) represents the decision and control quantity of UAV, and **r**(*·*) represents some uncertainties considered in the model.

It can be seen that the change law depends on two different kinds of decision and control vectors **u**(*·*) and **r**(*·*). Let **M** and **N** be two nonempty compact subsets of *ℝ*^*m*^ and *ℝ*^*p*^, respectively. Suppose that **A**:**=**{**u**:(0,*t*)⟶**M**}, **B**:**=**{**u**:(0,*t*)⟶**N**}, for each **z**(0) ∈ *ℝ*^d^ and (**u**,**r**) ∈ **A** × **B**, **z**=**z**_0_^**u**,**r**^ represents the relevant trajectory, which is defined as the system composed of equations (1)–(9).

Let **O** ⊂ *ℝ*^d^ be an open set, which is called “collision region.” All relative positions in the set are equivalent to collisions. The precise definition of the set will depend on the selection of dynamic state space. Here, the collision region **O** is regarded as an obstacle, and its complement **K=***ℝ*^d^/**O** represents the set of state constraints.

Different safety zones are defined as follows:

1. Set **W**_1_. It is defined as a subset of the initial position, so that for any control strategy, UAV cannot guarantee to avoid collision.
2. Set **W**_2_(*t*_*f*_). It is defined as the set of all initial states in *ℝ*^d^/**W**_1_, so that if there is no maneuver, there will be a risk that the system reaches region **W**_1_ before time *t*_*f*_.

## 4. Swarm Anticollision Game Decision and Control

### 4.1. Game Theory Model of Swarm Anticollision Problem

In order to analyze the security of systems with both control and disturbance, the worst-case method in antinatural game can be used. Disturbances are regarded as opponents of control and undermine security. For autonomous anticollision control, a game problem involving two parties is considered. One party is any member in the swarm, and the other party is each member adjacent to it. Here, the dynamic model of the relative position between each member adjacent to it and any member is

(35) $$\begin{array}{c} \dot{X}=f{}^{\prime }\left(X\left(t\right),u\left(t\right),r\left(t\right)\right), \end{array}$$

where **X** represents the state variable, **u** represents the control quantity of UAV, and **r** represents the uncertainty of the system, which plays the role of controlling the second player.

Meanwhile, the above formula meets the following conditions:

1. For each $\left(X,\dot{X},u,r\right)\in {\mathbb{R}}^{\text{d}}\times {\mathbb{R}}^{\text{d}}\times Μ\times N$, there is *L*_*f*_ > 0 such that $\left|f{}^{\prime }\left(X,u,r\right)-f{}^{\prime }\left(\dot{X},u,r\right)\right|\leq L_{f}\left|X-\dot{X}\right|$, where *L*_*f*_ is the Lipschitz constant
2. For each **X** ∈ *ℝ*^d^ and **r** ∈ **M**, *f*′(**X**, **M**, **r**) is a convex set of *ℝ*^d^

### 4.2. Solution of Decision and Control Strategy Set

As can be seen from Sections 3 and 3.1, the anticollision problem is described as a problem staying in a given closed set **K=***ℝ*^d^/**O**, and the autonomous anticollision problem is transformed into a game framework involving two parties. At this time, the set **W**_1_ can be described by the worst case of the game, which is that the first party player (UAV) wants to avoid the collision area **O**, or equivalent to keeping the system in the safe area **K** (through its own input **u**). The unexpected strategy set of player 1 (UAV) is defined as

(36) $$\begin{array}{c} \Gamma :\left\{u:B⟶A,\forall s\in \left[0,\infty \right],\left(r\left(\xi \right)=\tilde{r}\left(\xi \right),\forall \xi \in \right.\right.\\ \left.\left.\left[0,s\right]\right)\Rightarrow \left(u\left[r\right]\left(\xi \right)=u\left[\tilde{r}\right]\left(\xi \right),\forall \xi \in \left[0,s\right]\right)\right\}. \end{array}$$

Then, the selection of UAV control law is limited to the set Γ, and the victory domain of player 1 (UAV) is defined.

The victory domain of player 1: the set **V**_1_(**K**) of all initial positions *z*_0_. There is an unexpected strategy *F* ∈ Γ, which can ensure that all corresponding trajectories *z*_0_^**u**[**r**],**r**^(*t*) avoid collision set **O** for all ∈ and the allowable control **r** ∈ **B**. And **V**_1_(**K**) is

(37) $$\begin{array}{c} V_{1}\left(K\right)=\left\{z_{0}\in K|\exists F\in \Gamma ,\forall r\left(\cdot \right)\in B\right.,\\ \left.\forall t\geq 0,z_{0}^{u\left[r\right],r}\left(t\right)\in K\right\}. \end{array}$$

According to the definition, the two decision and control policy sets are

(38) $$\begin{array}{c} W_{1}=\frac{{\mathbb{R}}^{3}}{V_{1}\left(K\right)}, \end{array}$$

(39) $$\begin{array}{c} W_{2}\left(t_{f}\right)=\left\{z_{0}\in {\mathbb{R}}^{\text{d}},\exists r\left(\cdot \right)\in B,\exists s\in \left[0,t_{f}\right]\right., \end{array}$$

### 4.3. Swarm System Stability Analysis

This section analyzes the stability of swarm system based on linear feedback control theory. Taking the cohesion rule as an example, it is proved that each UAV member in the swarm system flies with the centroid of other UAVs in the swarm, and the swarm system will eventually reach a stable equilibrium state.

#### 4.3.1. Stability Analysis of Two UAV Members

The relative position relationship of the two UAV members is shown in Figure 2. The velocity vectors **V**_1_, **V**_2_ of the UAV are orthogonally decomposed along the sight distance line and the direction perpendicular to the sight distance line of the two UAV members, and the following can be obtained:

(40) $$\begin{array}{c} {\dot{R}}^{r}=V_{2}\cos\;\theta_{2}\cos\;\theta^{r}\cos\left(\psi_{2}-\psi^{r}\right)+V_{2}\sin\;\theta_{2}\sin\;\theta^{r} \end{array}$$

(41) $$\begin{array}{c} {\dot{\psi }}^{r}=\frac{V_{2}\cos\;\theta_{2}\sin\left(\psi_{2}-\psi^{r}\right)-V_{1}\cos\;\theta_{1}\sin\left(\psi_{2}-\psi^{r}\right)}{R^{r}\cos\;\theta^{r}}, \end{array}$$

(42) $$\begin{array}{c} {\dot{\theta }}^{r}=\frac{-V_{2}\cos\;\theta_{2}\sin\;\theta^{r}\cos\left(\psi_{2}-\psi^{r}\right)+V_{2}\sin\;\theta_{2}\cos\;\theta^{r}}{R^{r}}\\ +\frac{V_{1}\cos\;\theta_{1}\sin\;\theta^{r}\cos\left(\psi_{1}-\psi^{r}\right)-V_{1}\sin\;\theta_{1}\cos\;\theta^{r}}{R^{r}}, \end{array}$$

(43) $$\begin{array}{c} {\dot{\psi }}_{1}=\frac{-k_{1}\left(\psi_{1}-\psi^{r}\right)}{V_{1}\cos\;\theta_{1}}, \end{array}$$

(44) $$\begin{array}{c} {\dot{\theta }}_{1}=\frac{-k_{2}\left(\theta_{1}-\theta^{r}\right)}{V_{1}}, \end{array}$$

(45) $$\begin{array}{c} {\dot{\psi }}_{2}=\frac{k_{1}\left[\pi -\left(\psi_{2}-\psi^{r}\right)\right]}{V_{2}\cos\;\theta_{2}}, \end{array}$$

(46) $$\begin{array}{c} {\dot{\theta }}_{2}=\frac{k_{2}\left(-\theta_{2}-\theta^{r}\right)}{V_{1}}. \end{array}$$

Let *δψ*_1_=(*ψ*_1_ − *ψ*^*r*^), *δψ*_2_=(*ψ*_2_ − *ψ*^*r*^), select six state variables as *R*^*r*^, *δψ*_1_, *δψ*_2_, *θ*^*r*^, *θ*_1_, *θ*_2_, respectively, and linearize the above equations to obtain the following state equations:

(47) $$\begin{array}{c} \left[\begin{array}{c} {\dot{R}}^{r}\\ \delta {\dot{\psi }}_{1}\\ \delta {\dot{\psi }}_{2}\\ {\dot{\theta }}^{r}\\ {\dot{\theta }}_{1}\\ {\dot{\theta }}_{2} \end{array}\right]=\left[\begin{array}{cccccc} 0 & -V_{1} & -V_{2} & \text{0} & \text{0} & \text{0}\\ \frac{V_{1}+V_{2}}{{R^{r}}^{2}} & \frac{-k_{1}}{V_{1}} & \text{0} & \text{0} & \text{0} & \text{0}\\ \frac{V_{1}+V_{2}}{{R^{r}}^{2}} & \text{0} & \frac{-k_{1}}{V_{2}} & \text{0} & \text{0} & \text{0}\\ \text{0} & \text{0} & \text{0} & \text{0} & \frac{-V_{1}}{R^{r}} & \frac{V_{2}}{R^{r}}\\ \text{0} & \text{0} & \text{0} & \frac{-k_{2}}{V_{1}} & \frac{k_{2}}{V_{1}} & \text{0}\\ \text{0} & \text{0} & \text{0} & \frac{-k_{2}}{V_{2}} & \text{0} & \frac{-k_{2}}{V_{2}} \end{array}\right]\left[\begin{array}{c} R^{r}\\ \delta \psi_{1}\\ \delta \psi_{2}\\ \theta^{r}\\ \theta_{1}\\ \theta_{2} \end{array}\right]. \end{array}$$

In order to simplify the calculation, let *V*_1_=*V*_2_=*V* and *k*_1_=*k*_2_=*k*; according to the Laplace transform and the maximum value theory, the state of the equilibrium point is

(48) $$\begin{array}{c} R^{r}=\frac{2V^{2}}{\left(k\pi /2\right)},\\ \delta \psi_{1}=\frac{-\pi }{2},\\ \delta \psi_{2}=\frac{\pi }{2},\\ \theta^{r}=0,\\ \theta_{1}=0,\\ \theta_{2}=0. \end{array}$$

Let *V*=*x*_1_, 2*V*/*R*^*r*^^2^=*x*_2_, *k*/*V*=*x*_3_, *V*/*R*^*r*^=*x*_4_, then the characteristic equation becomes

(49) $$\begin{array}{c} \det\left(\lambda I-A\right)=0. \end{array}$$

The obtained eigenvalues are

(50) $$\begin{array}{c} \lambda =-x_{3},-x_{3},-\frac{1}{2}x_{3}\pm \sqrt{{x_{3}}^{2}-8x_{1}x_{2}},-\frac{1}{2}x_{3}\pm \sqrt{{x_{3}}^{2}-8x_{3}x_{4}}. \end{array}$$

Because *x*_1_, *x*_2_, *x*_3_, *x*_4_ > 0, *x*_3_^2^=(*k*/*V*)^2^ and 8*x*_1_*x*_2_=*π*^2^(*k*/*V*)^2^, 8*x*_3_*x*_4_=2*π*(*k*/*V*)^2^, we have 8*x*_1_*x*_2_ > *x*_3_^2^, 8*x*_3_*x*_4_ > *x*_3_^2^, and the eigenvalues of the characteristic equation are negative real numbers. Therefore, ∀*k*, *V*, the dual computer system composed of two UAV members is stable.

#### 4.3.2. Stability Analysis of *n* UAV Members

Under the cohesion rule, the *i*-th UAV member in the swarm system follows the centroid motion of the other (*n* − 1) UAV members. Here, the average centroid of these (*n* − 1) UAV members is regarded as a virtual UAV member, and its track deflection angle and track inclination angle are expressed as

(51) $$\begin{array}{c} \psi_{i_{n-1}}=\left(\frac{1}{n-1}\right)\sum_{j=1,j\neq i}^{n}\left(\psi_{j}\right), \end{array}$$

(52) $$\begin{array}{c} \theta_{i_{n-1}}=\left(\frac{1}{n-1}\right)\sum_{j=1,j\neq i}^{n}\left(\theta_{j}\right). \end{array}$$

At this time, the line of sight vector *R*_*ii*_*n*−1__^*r*^, expected track deflection angle *ψ*_*ii*_*n*−1__^*r*^, and track inclination angle *θ*_*ii*_*n*−1__^*r*^ are, respectively,

(53) $$\begin{array}{c} R_{ii_{n-1}}^{r}=\left(\frac{1}{n-1}\right)\sum_{j=1,j\neq i}^{n}\left(R_{ij}^{r}\right), \end{array}$$

(54) $$\begin{array}{c} \psi_{ii_{n-1}}^{r}=\left(\frac{1}{n-1}\right)\sum_{j=1,j\neq i}^{n}\left(\psi_{ij}^{r}\right), \end{array}$$

(55) $$\begin{array}{c} \theta_{ii_{n-1}}^{r}=\left(\frac{1}{n-1}\right)\sum_{j=1,j\neq i}^{n}\left(\theta_{ij}^{r}\right). \end{array}$$

Then, the speed acceleration term is

(56) $$\begin{array}{c} \kappa_{\psi i}=-k\left(\psi_{i}-\psi_{ii_{n-1}}^{r}\right), \end{array}$$

(57) $$\begin{array}{c} \kappa_{\theta i}=-k\left(\theta_{i}-\theta_{ii_{n-1}}^{r}\right). \end{array}$$

Combining Equations (56) and (57) with Equations (4) and (5), respectively, we have

(58) $$\begin{array}{c} {\dot{\psi }}_{i}=\frac{-k\left(\psi_{i}-\psi_{ii_{n-1}}^{r}\right)}{V\;\cos\;\theta_{i}}, \end{array}$$

(59) $$\begin{array}{c} {\dot{\theta }}_{i}=\frac{-k\left(\theta_{i}-\theta_{ii_{n-1}}^{r}\right)}{V}. \end{array}$$

Similarly, it can be considered that the virtual point of (*n* − 1) UAV member follows the flight of the *i*-th UAV member, and the track deflection angular velocity acceleration term is expressed as

(60) $$\begin{array}{c} \kappa_{\psi i_{n-1}}=\left(\frac{1}{n-1}\right)\sum_{j=1,j\neq i}^{n}\kappa_{\psi j}=\left(\frac{1}{n-1}\right)\sum_{j=1,j\neq i}^{n}-k\left(\psi_{j}-\psi_{jj_{n-1}}^{r}\right)\\ =\left(\frac{k}{n-1}\right)\left(-\sum_{j=1,j\neq i}^{n}\psi_{j}+\sum_{j=1,j\neq i}^{n}\psi_{jj_{n-1}}^{r}\right). \end{array}$$

Here

(61) $$\begin{array}{c} \sum_{j=1,j\neq i}^{n}\psi_{jj_{n-1}}^{r}=\left(\psi_{11_{n-1}}^{r}+\psi_{22_{n-1}}^{r}+\cdots +\psi_{\left(i-1\right){\left(i-1\right)}_{n-1}}^{r}+\psi_{\left(i+1\right){\left(i+1\right)}_{n-1}}^{r}+\cdots +\psi_{nn_{n-1}}^{r}\right),\\ =\left(\frac{1}{n-1}\right)\left(\left(\psi_{12}^{r}+\psi_{13}^{r}+\cdots +\psi_{1n}^{r}\right)+\left(\psi_{21}^{r}+\psi_{23}^{r}\cdots +\psi_{2n}^{r}\right)+\cdots \right.\\ +\left(\psi_{\left(i+1\right)1}^{r}+\psi_{\left(i+1\right)2}^{r}+\cdots +\psi_{\left(i+1\right)\left(i-2\right)}^{r}+\psi_{\left(i-1\right)i}^{r}+\cdots +\psi_{\left(i-1\right)n}^{r}\right)\\ +\cdots +\left(\psi_{\left(i+1\right)1}^{r}+\psi_{\left(i+1\right)2}^{r}+\cdots \cdot +\psi_{\left(i+1\right)i}^{r}+\psi_{\left(i+1\right)\left(i-2\right)}^{r}+\cdots \right.\\ \left.\left.+\psi_{\left(i+1\right)n}^{r}\right)+\cdots +\left(\psi_{n1}^{r}+\psi_{n2}^{r}+\cdots +\psi_{n\left(n-1\right)}^{r}\right)\right). \end{array}$$

According to the relative position relationship of UAV, it can be seen that *ψ*_*ij*_^*r*^=*π* − *ψ*_*ji*_^*r*^; then,

(62) $$\begin{array}{c} \sum_{j=1,j\neq i}^{n}\psi_{jj_{n-1}}^{r}=\pi \left(n-1\right)+\sum_{j=1,j\neq i}^{n}\psi_{ij}^{r}. \end{array}$$

Substituting equation (62) into equation (60), the following can be obtained:

(63) $$\begin{array}{c} \kappa_{\psi i_{n-1}}=k\left\{\pi -\left(\frac{1}{n-1}\sum_{j=1,j\neq i}^{n}\psi_{j}-\frac{1}{n-1}\sum_{j=1,j\neq i}^{n}\psi_{ij}^{r}\right)\right\}. \end{array}$$

It can be obtained from equations (50) and (54) that

(64) $$\begin{array}{c} \kappa_{\psi i_{n-1}}=k\left(\pi -\left(\psi_{i_{n-1}}-\psi_{ii_{n-1}}^{r}\right)\right). \end{array}$$

Simultaneously equation (62) and equation (4) can obtain

(65) $$\begin{array}{c} {\dot{\psi }}_{i_{n-1}}=\frac{k\left(\pi -\left(\psi_{i_{n-1}}-\psi_{ii_{n-1}}^{r}\right)\right)}{V\;\cos\;\theta_{i_{n-1}}}. \end{array}$$

Similarly, the track inclination velocity acceleration term is expressed as

(66) $$\begin{array}{c} \kappa_{\theta i_{n-1}}=\left(\frac{1}{n-1}\right)\sum_{j=1,j\neq i}^{n}\kappa_{\theta j},\\ =\left(\frac{1}{n-1}\right)\sum_{j=1,j\neq i}^{n}-k\left(\theta_{j}-\theta_{jj_{n-1}}^{r}\right),\\ =\left(\frac{k}{n-1}\right)\left(-\sum_{j=1,j\neq i}^{n}\theta_{j}+\sum_{j=1,j\neq i}^{n}\theta_{jj_{n-1}}^{r}\right), \end{array}$$

where

(67) $$\begin{array}{c} \sum_{j=1,j\neq i}^{n}\theta_{jj_{n-1}}^{r}=\left(\theta_{11_{n-1}}^{r}+\theta_{22_{n-1}}^{r}+\cdots +\theta_{\left(i-1\right){\left(i-1\right)}_{n-1}}^{r}+\theta_{\left(i+1\right){\left(i+1\right)}_{n-1}}^{r}+\cdots +\theta_{nn_{n-1}}^{r}\right),\\ =\left(\frac{1}{n-1}\right)\left(\left(\theta_{12}^{r}+\theta_{13}^{r}+\cdots +\psi_{1n}^{r}\right)+\left(\theta_{21}^{r}+\theta_{23}^{r}\cdots +\theta_{2n}^{r}\right)+\cdots \right.\\ +\left(\theta_{\left(i+1\right)1}^{r}+\theta_{\left(i+1\right)2}^{r}+\cdots +\theta_{\left(i+1\right)\left(i-2\right)}^{r}+\theta_{\left(i-1\right)i}^{r}+\cdots +\theta_{\left(i-1\right)n}^{r}\right)\\ +\cdots +\left(\theta_{\left(i+1\right)1}^{r}+\theta_{\left(i+1\right)2}^{r}+\cdots \cdot +\theta_{\left(i+1\right)i}^{r}+\theta_{\left(i+1\right)\left(i-2\right)}^{r}+\cdots \right.\\ \left.\left.+\theta_{\left(i+1\right)n}^{r}\right)+\cdots +\left(\theta_{n1}^{r}+\theta_{n2}^{r}+\cdots +\theta_{n\left(n-1\right)}^{r}\right)\right). \end{array}$$

According to the relative position relationship of UAV, it can be seen that *θ*_*ij*_^*r*^=−*θ*_*ji*_^*r*^; then,

(68) $$\begin{array}{c} \sum_{j=1,j\neq i}^{n}\theta_{jj_{n-1}}^{r}=-\sum_{j=1,j\neq i}^{n}\theta_{ij}^{r}. \end{array}$$

Substituting equation (68) into equation (66), the following can be obtained:

(69) $$\begin{array}{c} \kappa_{\theta i_{n-1}}=\frac{k}{n-1}\left(-\sum_{j=1,j\neq i}^{n}\theta_{j}-\sum_{j=1,j\neq i}^{n}\theta_{ij}^{r}\right). \end{array}$$

It can be obtained from equations (52) and (55) that

(70) $$\begin{array}{c} \kappa_{\theta i_{n-1}}=-k\left(\theta_{i_{n-1}}+\theta_{ii_{n-1}}^{r}\right). \end{array}$$

Simultaneously equation (70) and equation (5) can obtain

(71) $$\begin{array}{c} {\dot{\theta }}_{i_{n-1}}=\frac{-k\left(\theta_{i_{n-1}}+\theta_{ii_{n-1}}^{r}\right)}{V}. \end{array}$$

According to equations (40)–(46), the virtual point of (*n* − 1) UAV members is regarded as the second member of the two UAV members; that is, *ψ*_2_,  *θ*_2_ is replaced by *ψ*_*i*_*n*−1__,  *θ*_*i*_*n*−1__, and the sight distance vector *R*^*r*^, expected track deflection angle, and track inclination angle *ψ*^*r*^,  *θ*^*r*^ are replaced by *R*_*ii*_*n*−1__^*r*^ and *ψ*_*ii*_*n*−1__^*r*^,  *θ*_*ii*_*n*−1__^*r*^, respectively. The forms of equations (58), (59), (65) and (70), (47) are similar to equations (48)–(53) established by two UAV members in the sight distance direction. Therefore, the stability of two UAV members in the swarm system can be analyzed and proved by the stability of two UAV members. According to Section 4.1, the swarm system composed of *n* UAV members has a stable equilibrium state; that is, the swarm system is stable.

## 5. Simulation Experiment and Verification

In order to facilitate the result analysis and discussion, the simulation verification of UAV swarm flight and cooperative avoidance in two-dimensional plane is mainly carried out. Without losing generality, the simulation scenario is set as avoidance between two swarm systems. For one swarm, the other swarm is collision threat. Both swarm systems adopt the autonomous cooperative control method of flight and avoidance proposed in this paper. In this scenario, the following three simulation experiments are carried out.

### 5.1. Simulation 1: Swarm System Avoidance Process

The overall evasion mechanism and member evasion mechanism are used to simulate the evasion process of two UAV swarm systems in two-dimensional space. The swarms are in the two-dimensional horizontal plane, and the avoidance decision mainly depends on the change of track deflection angle of UAV members. The speed of UAV members is constant as 20*m*/*s*, and *s*_min_=60*m*, *s*_1_=150*m*, and *s*_2_=60*m*. The available detection distance of airborne sensors is set to a fixed value *ρ*=600*m*, and the other two are *ρ*_*c*_=400*m* and *ρ*_*e*_=600*m*. The initial track deflection angles of the two swarm systems are *ψ*_1_=0°, *ψ*_2_=180°. The dynamic characteristics of UAV and the constraints are roll angle −20° ≤ *ϕ*_c_ ≤ 20°, overload in pitch plane *n*_*y*_ ≤ 2*g*, overload in yaw plane *n*_*z*_ ≤ 4*g*, and turning radius *r*_*d*_ ≥ 200*m*. When the swarm system flies normally, the initial value of the weight corresponding to each flight rule is

(72) $$\begin{array}{c} \tau_{i_{M}}=0.55,\tau_{i_{F}}.\\ =0.22,\tau_{i_{I}},\\ =0.78,\tau_{i_{S}},\\ =0.55,\tau_{i_{A}},\\ =0.42,\tau_{i_{E}},\\ =0. \end{array}$$

If the swarm system detects external UAV members, under the overall and member avoidance mechanism, the weights change to, respectively,

(73) $$\begin{array}{c} \tau_{i_{M}}{}^{\prime }=0.55,\tau_{i_{F}}{}^{\prime },\\ =0.22,\tau_{i_{I}}{}^{\prime },\\ =0.38,\tau_{i_{S}}{}^{\prime },\\ =0.55,\tau_{i_{A}}{}^{\prime },\\ =0.42,\tau_{i_{E}}{}^{\prime },\\ =0.55,\\ \tau_{i_{M}}{}^{\prime \prime }=0.30,\tau_{i_{F}}{}^{\prime \prime },\\ =0.30,\tau_{i_{I}}{}^{\prime \prime },\\ =0.38,\tau_{i_{S}}{}^{\prime \prime },\\ =0.55,\tau_{i_{A}}{}^{\prime \prime },\\ =0.42,\tau_{i_{E}}{}^{\prime \prime },\\ =0.55. \end{array}$$

The avoidance process of UAV swarm is shown in Figures 3 and 4. The flight track of swarm 1 is represented by blue line and that of swarm 2 is represented by red line. During the avoidance process of the swarm system, the variation curves of the minimum distance *R*_min_ between UAV members and the maximum distance d_max_ from all UAV members to the swarm centroid are shown in Figure 5(a) and 5(b), respectively.

From the simulation 1 experimental results, it can be seen that under the action of basic flight rules, UAV swarm can maintain stable flight in a certain formation and can realize formation reconstruction after evasion. Under the action of overall evasion mechanism and member evasion mechanism, the swarm system can complete evasion and realize safe flight. The difference between the two mechanisms is that in the overall mechanism, the variation of UAV track deflection angle relative to the initial flight direction is relatively large; that is, the overall track cost is high. In the member mechanism, the overall change of UAV track deflection angle is small, but the change rate is large, and the avoidance process is more complex.

### 5.2. Simulation 2: The Influence of Flight Rule Weight on the Stable Scale of the Swarm System

The influence of several flight rule weight coefficients *τ*_*M*_, *τ*_*I*_, *τ*_*S*_ on the stable scale of swarm system is studied. First, make the weight of the self-guidance rule constant *τ*_*I*_=0.6, and the weight of the dispersion rule takes values *τ*_*S*_=0.2, *τ*_*S*_=0.4, *τ*_*S*_=0.6, respectively. The weight of the cohesion rule *τ*_*M*_ changes from 0.1 to 1.0. When the swarm system is stable, the scale changes with the weight of the cohesion rule, as shown in Figure 6(a). Then, let the weight of the dispersion rule be a constant value *τ*_*S*_=0.4, and the weight of the self-guidance rule takes values *τ*_*I*_=0.3, *τ*_*I*_=0.5, *τ*_*I*_=0.7, respectively. The weight of the cohesion rule *τ*_*M*_ changes from 0.1 to 1.0. When the swarm system is stable, the scale changes with the weight of the cohesion rule, as shown in Figure 6(b).

From the simulation 2 experimental results in Figure 6(a), it can be seen that the change trend of the scale of the swarm system is as follows: first, it decreases with the increase of the weight of the cohesion rule *τ*_*M*_ and then increases with the increase of *τ*_*M*_. This is because the cohesion within the swarm system is obvious at the beginning, and the stability of the swarm system gradually decreases with the continuous increase of *τ*_*M*_. As can be seen from Figure 6(b), the scale of the swarm system has a similar change trend and increases with the increase of the weight of the self-guidance rule *τ*_*I*_, because the cohesion decreases with the increase of *τ*_*I*_. It can be seen that the value of *τ*_*M*_ between 0.2 ~ 0.4 is more appropriate for the small scale and stability of the system.

### 5.3. Simulation 3: Real-Time Performance of Evasion Control

This paper discusses the real-time performance of swarm system evasion control method and compares it with MPC algorithm, in which MPC algorithm is proposed in reference [17]. In the two algorithms, the simulation scene settings are the same, and they are implemented in Visual *C*++ 6.0 and MATLAB R2021a environment. The computer is configured as Intel Core i5 processor, main frequency 3.10 GHz, memory 8 G, and 32-bit operating system. After multiple simulations, the average running time of the algorithm is shown in Figure 7.

It can be seen from the simulation 3 experimental results that the running time of MPC method increases exponentially with the increase of the number of formation UAVs. When the number of UAVs is large, the calculation efficiency is greatly reduced and the running time of the algorithm is long. The running time of the overall mechanism and member mechanism in the swarm algorithm increases slowly with the increase of the number of UAVs in the swarm. When the number of UAVs in the swarm is no more than 10, the execution time of the algorithm is within 25 ms, which can meet the needs of online real-time control.

## 6. Conclusions

In this paper, a cognitive game method is used to study the anticollision cooperative decision-making and control of UAV swarms, and the method is used to simulate the flight and avoidance process between UAV swarms. The basic flight behavior rules of UAV swarm are designed. Under the action of these rules, UAV swarm can realize normal flight and formation reconstruction. Aiming at the problem of anticollision, two anticollision mechanisms, named whole and member mechanism, are put forward. At the same time, a cognitive security domain facing swarm anticollision is constructed. On this basis, the game theory model of swarm anticollision problem is established, and the solution method of swarm anticollision game decision and control strategy is designed. Finally, the stability of UAV swarm system using the above method is analyzed. Simulation results show that compared with the traditional MPC method, the swarm control proposed in this paper is simpler and more efficient.

## Figures and Tables

**Figure 1:** Geometric parameters of a single UAV member.

**Figure 2:** Relative geometric parameters of two UAV members.

**Figure 3:** Swarm avoidance process under the overall mechanism. (a) *t*=25*s*. (b) *t*=50*s*. (c) *t*=75*s*. (d) *t*=100*s*.

**Figure 4:** Swarm avoidance process under membership mechanism. (a) *t*=25*s*. (b) *t*=50*s*. (c) *t*=75*s*. (d) *t*=100*s*.

**Figure 5:** Variation curves of *R*_min_ and d_max_. (a) Overall mechanism. (b) Membership mechanism.

**Figure 6:** Influence of weight change of flight rules on system scale. (a) *τ*_*I*_=0.6, *τ*_*S*_=0.2, 0.4, 0.6. (b) *τ*_*S*_=0.4, *τ*_*I*_=0.3, 0.5, 0.7.

**Figure 7:** Comparison of average running time of algorithm.

## Data Availability

The data used to support the findings of this study are included within the article.
